# Staying awake to stay alive: A circuit controlling starvation-induced waking

**DOI:** 10.1371/journal.pbio.3000199

**Published:** 2019-03-27

**Authors:** Krishna Melnattur, Paul Shaw

**Affiliations:** Department of Neuroscience, Washington University School of Medicine, St. Louis, Missouri, United States of America

## Abstract

The balance of sleep and wake is plastic and changes to meet environmental demands. Mechanisms that allow an animal to suppress sleep and maintain waking in potentially adverse situations could serve adaptive functions in evolution. The fruit fly, *Drosophila melanogaster*, is well poised as a system in which to explore these questions. The environment changes sleep and wake in flies, e.g., starvation induces waking in *Drosophila* as it does in many animals. Further, the sophisticated neurobiological toolkit available to *Drosophila* researchers gives the fly a great advantage as a system to investigate the precise neurobiological mechanisms underlying these adaptive changes. In a paper in this issue of *PLOS Biology*, Yurgel and colleagues elegantly exploit the advantages of the *Drosophila* model to map starvation-induced wakefulness to a single pair of peptidergic neurons and their partners.

## Abstract 2

Which neural sites mediate the effects of environmental changes on sleep and waking? This Primer explores a recent elegant study in fruit flies which localizes the effects of starvation-induced wakefulness to a single pair of peptidergic neurons.

Sleep duration is modulated by both genetic and environmental factors [1,2]. It has been suggested that genetic modifiers that allow individuals to maintain waking in dangerous conditions would serve such an important adaptive value that they would be preserved during the course of evolution [3]. If this is true, identifying genes and circuits that influence waking in adverse environments may have relevance for understanding genetic variation in sleep duration in humans and potentially unexplored risk factors for human sleep disorders. Indeed, the genetic model organism *D*. *melanogaster* is well suited for dissecting the genes and circuits underlying adaptive waking [4]. In this issue of *PLOS Biology*, Yurgel and colleagues [5] have mapped starvation-induced wakefulness to a single pair of peptidergic neurons and their downstream targets. Moreover, they have identified AMP-activated protein kinase (AMPK) as the critical signaling molecule.

In a previous study, Murakami and colleagues [6] identified transilin, a conserved RNA/DNA-binding protein, as a key molecular mediator of adaptive waking during starvation. Although the authors localized the effects of transilin to neurons expressing the neuropeptide leukokinin (Lk), the precise neurons remained unclear. Lk is expressed in approximately 30 neurons in the adult fly central nervous system (CNS), organized in four distinct clusters (Fig 1): one row of cells in the abdominal ganglion (ABLK), a pair of neurons in the subesophageal zone in the brain (SELK), two pairs of anterior-located neurons (ALK), and a single pair of neurons in the lateral horn (LHLK). The leukokinin receptor (Lkr), in contrast, is more widely expressed in the CNS and peripheral tissues. *Lk* mutants impact a large and diverse set of physiological systems, raising the possibility that each different site of *Lk* expression would individually control specific functions.

**Fig 1:** Schematic depicting the various Lk-expressing cells in the adult fly CNS. Lk is expressed in approximately 30 neurons in the adult fly CNS, distributed in four distinct clusters, that appear to subserve different functions. The ABLK were recently implicated in maintenance of water homeostasis, presumably by acting on Lkr in peripheral tissues. In the brain, Lk signaling between the LHLK and LkrFB has been previously implicated in the expression of circadian activity and postprandial sleep. In a study in this issue of *PLOS Biology*, Yurgel and colleagues elegantly demonstrate that Lk signaling between LHLK and LkrPI is required for the expression of starvation-induced wakefulness. ABLK, abdominal ganglion Lk; CNS, central nervous system; LHLK, lateral horn Lk; Lk, leukokinin; Lkr, leukokinin receptor; LkrFB, fan-shaped body projecting Lkr neurons; LkrPI, Lkr-expressing neurons in the pars intercerebralis.

To map the relevant sites of *Lk* function, Yurgel and colleagues [5] used an impressive *Drosophila* toolkit including clustered regularly interspaced short palindromic repeats (CRISPR) gene editing and an innovative laser-ablation technique. CRISPR gene editing was used to generate novel GAL4 lines for *Lk* and *Lkr*, wherein GAL4 was inserted into the native gene locus. This strategy allows for both monitoring and manipulating *Lk* and *Lkr*-expressing cells (by crossing the GAL4 lines to various upstream activating sequence (UAS) effector lines) and for examining consequences of *Lk* loss of function (as inserting GAL4 also disrupts the native gene locus). Using cell type–specific knockdown of gene function with RNA interference (RNAi) and cell type–specific rescue, they were able to show that *Lk* function in the LHLK (Fig 1) is necessary and sufficient for starvation-induced wakefulness and hyperactivity. Blocking synaptic transmission from the LHLK neurons phenocopied the data from the Lk loss-of-function experiments.

These results were confirmed in an elegant ablation experiment. Specifically, laser ablation of the LHLK but not the ALK (Fig 1) abolished the ability of starvation to induce wakefulness. These functional experiments demonstrated that the output of the LHLK is required for the response to starvation and suggested the possibility that the LHLK neurons are activated by starvation. Calcium imaging of the LHLK neurons confirmed that these neurons were indeed activated following starvation. Together, these data demonstrate that a single pair of *Lk* neurons, the LHLK neurons (Fig 1), are critical for behavioral response to starvation.

But which of the many Lkr-expressing cells are required? As mentioned, the Lkr is expressed broadly throughout the brain, including a set of neurons that project into the dorsal fan-shaped body, an important sleep-promoting structure in the *Drosophila* brain. The authors address this question by knocking down Lkr with RNAi and by blocking synaptic transmission in subsets of Lkr-expressing cells. These independent sets of experiments localized the downstream circuit components of adaptive waking to the LkrPI neurons (Fig 1) that are part of the pars intercerebralis (PI) and not the previously identified Lkr neurons that project to the fan-shaped body (LkrFB neurons). The PI is an important neuroendocrine center in the fly brain, previously implicated in a range of behaviors from courtship and ethanol sensitivity to circadian locomotor rhythms and sleep [7–10].

This paper is the latest chapter in a growing body of work from a number of groups that have, of late, begun to dissect the roles of specific Lk and Lkr-expressing cells in regulating many aspects of physiology and behavior. For example, a recent study in *PLOS Genetics* found that *Lk* signaling regulates water homeostasis [11]. Importantly, the authors mapped the sites of *Lk* action to the ABLK as well as peripheral tissues, including the renal pads and malphigian tubules [11]. Moreover, Cavey and colleagues identified a role of Lk and Lkr in behavioral locomotor rhythms [12]. In this study, the authors identified Lk as a regulator of behavioral rhythms in a neuropeptide screen. Since neither Lk nor Lkr-expressing cells expressed components of the molecular clock, they suggest that Lk circuits represent outputs of the clock. By examining calcium activity of subsets of Lk neurons, they found that the LHLK and Lkr cells that project to the LkrFB exhibit circadian rhythmicity in their calcium activity. Together, these data implicate the LHLK–LkrFB microcircuit in the control of circadian rhythms. Independently, Murphy and colleagues [13], while examining the mechanisms of postprandial sleep, determined that the expression of this phenomenon was dependent on Lk signaling and required the activity of the LkrFB neurons.

To fully appreciate the importance of Yurgel and colleagues’ contribution to the field, one must acknowledge that the broader set of Lk neurons, while showing many similar features, are in fact quite heterogeneous. Without mapping the precise pair of neurons responsible for starvation-induced waking, it would not be possible for future studies to fully dissect the functional role of this system with certainty. Indeed, manipulations that impact the entire set of neurons would produce confounding results, and it would be difficult, if not impossible, to disentangle the interaction between these competing physiological processes or how they modulate adaptive behavior in an ever-changing environment. The importance of taking the time to map the precise neurons involved in a phenotype is a significant advance. This conclusion is reinforced by a study demonstrating that a single pair of dopaminergic neurons is important for sleep regulation [14]. Indeed, while the role of dopamine in waking has been well understood for decades in mammals and flies [15,16], mapping the precise pair of dopaminergic neurons that control sleep in flies has been, and continues to be, instrumental in advancing our understanding of sleep drive [17]. Although the murine toolkit is becoming increasingly precise, it is not yet possible to gain genetic access to such small subsets of unique neurons. As a consequence, these findings highlight the continued importance of the *Drosophila* toolkit for truly dissecting circuit function.

## Abbreviations

ABLK: abdominal ganglion Lk
ALK: anterior-located Lk
CNS: central nervous system
CRISPR: clustered regularly interspaced short palindromic repeats
LHLK: lateral horn Lk
Lk: leukokinin
Lkr: leukokinin receptor
LkrFB: fan-shaped body projecting Lkr neurons
LkrPI: Lkr-expressing neurons in the pars intercerebralis
RNAi: RNA interference
SELK: subesophageal zone Lk
UAS: upstream activating sequence

## References

[1] UrryE, LandoltHP. Adenosine, caffeine, and performance: from cognitive neuroscience of sleep to sleep pharmacogenetics. Current topics in behavioral neurosciences. 2015;25:331–66. 10.1007/7854_2014_274 24549722

[2] ZhangL, FuYH. The molecular genetics of human sleep. The European journal of neuroscience. 2018.10.1111/ejn.14132PMC638944330144347

[3] WillieJT, ChemelliRM, SintonCM, YanagisawaM. To eat or to sleep? Orexin in the regulation of feeding and wakefulness. Annual review of neuroscience. 2001;24:429–58. 10.1146/annurev.neuro.24.1.429 11283317

[4] DonleaJ, LeahyA, ThimganMS, SuzukiY, HughsonBN, SokolowskiMB, et al Foraging alters resilience/vulnerability to sleep disruption and starvation in Drosophila. Proc Natl Acad Sci U S A. 2012;109(7):2613–8. 10.1073/pnas.1112623109 22308351PMC3289360

[5] YurgelME, KakadP, ZandawalaM, NässelDR, GodenschwegeTA, KeeneAC. A single pair of leucokinin neurons are modulated by feeding state and regulate sleep-metabolism interactions. PLoS Biol. 2019: 17(2): e2006409 10.1371/journal.pbio.200640930759083PMC6391015

[6] MurakamiK, YurgelME, StahlBA, MasekP, MehtaA, HeidkerR, et al translin Is Required for Metabolic Regulation of Sleep. Curr Biol. 2016;26(7):972–80. 10.1016/j.cub.2016.02.013 27020744PMC4846466

[7] SakaiT, WatanabeK, OhashiH, SatoS, InamiS, ShimadaN, et al Insulin-producing cells regulate the sexual receptivity through the painless TRP channel in Drosophila virgin females. PLoS ONE. 2014;9(2):e88175 10.1371/journal.pone.0088175 24505416PMC3913769

[8] DevineniAV, EddisonM, HeberleinU. The novel gene tank, a tumor suppressor homolog, regulates ethanol sensitivity in Drosophila. J Neurosci. 2013;33(19):8134–43. 10.1523/JNEUROSCI.3695-12.2013 23658154PMC3865512

[9] CavanaughDJ, GeratowskiJD, WooltortonJR, SpaethlingJM, HectorCE, ZhengX, et al Identification of a circadian output circuit for rest:activity rhythms in Drosophila. Cell. 2014;157(3):689–701. 10.1016/j.cell.2014.02.024 24766812PMC4003459

[10] FoltenyiK, GreenspanRJ, NewportJW. Activation of EGFR and ERK by rhomboid signaling regulates the consolidation and maintenance of sleep in Drosophila. Nat Neurosci. 2007;10(9):1160–7. 10.1038/nn1957 17694052

[11] ZandawalaM, YurgelME, TexadaMJ, LiaoS, RewitzKF, KeeneAC, et al Modulation of Drosophila post-feeding physiology and behavior by the neuropeptide leucokinin. PLoS Genet. 2018;14(11):e1007767 10.1371/journal.pgen.1007767 30457986PMC6245514

[12] CaveyM, CollinsB, BertetC, BlauJ. Circadian rhythms in neuronal activity propagate through output circuits. Nat Neurosci. 2016;19(4):587–95. 10.1038/nn.4263 26928065PMC5066395

[13] MurphyKR, DeshpandeSA, YurgelME, QuinnJP, WeissbachJL, KeeneAC, et al Postprandial sleep mechanics in Drosophila. Elife. 2016;5.10.7554/eLife.19334PMC511988727873574

[14] LiuQ, LiuS, KodamaL, DriscollMR, WuMN. Two dopaminergic neurons signal to the dorsal fan-shaped body to promote wakefulness in Drosophila. Curr Biol. 2012;22(22):2114–23. 10.1016/j.cub.2012.09.008 23022067PMC3505250

[15] AndreticR, van SwinderenB, GreenspanRJ. Dopaminergic modulation of arousal in Drosophila. Curr Biol. 2005;15(13):1165–75. 10.1016/j.cub.2005.05.025 16005288

[16] JonesBE. Neurobiology of waking and sleeping. Handbook of clinical neurology / edited by PJ Vinken and GW Bruyn. 2011;98:131–49.10.1016/B978-0-444-52006-7.00009-5PMC554810621056184

[17] PimentelD, DonleaJM, TalbotCB, SongSM, ThurstonAJ, MiesenbockG. Operation of a homeostatic sleep switch. Nature. 2016;536(7616):333–7. 10.1038/nature19055 27487216PMC4998959

